The article "Prediction of Fetal Growth Restriction for Fetal Umbilical Arterial/Venous Blood Flow Index Evaluated by Ultrasonic Doppler under Intelligent Algorithm" was published in 2022. Journal: Comput Math Methods Med.

# Prediction of Fetal Growth Restriction for Fetal Umbilical Arterial/Venous Blood Flow Index Evaluated by Ultrasonic Doppler under Intelligent Algorithm

**DOI:** 10.1155/2022/7451185

**Published:** 2022-05-19

**Authors:** Xinying Yu, Ye Yao, Dan Wang, Jiani Tang, Jing Lu

**Affiliations:** ^1^Department of Obstetrics, The Affiliated Changzhou No.2 People's Hospital of Nanjing Medical University, Changzhou, 213004 Jiangsu, China; ^2^Department of Ultrasound, The Affiliated Changzhou No.2 People's Hospital of Nanjing Medical University, Changzhou, 213004 Jiangsu, China

## Abstract

The empirical wavelet transform (EWT) algorithm was applied in ultrasound to explore the predictive value for fetal growth restriction (FGR) in fetal arteriovenous indexes. 142 pregnant women who received prenatal ultrasonic examination and delivered were selected. They were classified into control group and FGR group. There were 102 patients with normal pregnancy in the control group, and 40 patients with delayed fetal growth in the FGR group. The extended triple collocation (ETC) algorithm was employed to divide the Fourier spectrum of signals adaptively, and the constructed small filter banks were classified into corresponding intervals. The instantaneous frequency was analyzed, and the arterial blood flow indexes of the two groups were compared. The results showed that the time-frequency analysis method under EWT had lower normalization error and higher accuracy. The inner diameter and cross-sectional area of FGR were remarkably smaller than those of the control group, and the differences were statistically significant (*P* < 0.05). There were no significant differences in mean blood flow and mean blood velocity between the control group and FGR group (*P* > 0.05). The arterial blood flow parameters of the systolic flow velocity (VS) and the diastolic flow velocity (VD) in the FGR group were notably lower than those in the control group, and the differences were significant (*P* < 0.05). In conclusion, the frequency principal component extracted by EWT algorithm was less disturbed by noise, which could accurately and effectively evaluate fetal arteriovenous blood flow indexes and predict FGR.

## 1. Introduction

Fetal growth restriction (FGR), known as intrauterine growth restriction, is defined as an abnormal fetal size that has not reached the growth potential in utero and is below the 10^th^ percentile of normal weight for the age [1, 2]. The incidence of FGR in China is 6.39%, the mortality rate is about 6-10 times of that of normal birth, and 50% of the perinatal infants has intrauterine hypoxia at birth. The umbilic-portal vein system is the only feeding route for the fetus. The increase in oxygen demand is accompanied by an increase in venous blood flow, with only about 43% of the venous blood flowing into the venous duct during the third trimester of pregnancy [3–5]. Early treatment and enhanced diagnosis of FGR is a crucial measure to reduce fetal morbidity. FGR is closely related to fetal intrauterine ischemia and hypoxia and ultimately affects the outcome of fetal birth [6].

The article "Prediction of Fetal Growth Restriction for Fetal Umbilical Arterial/Venous Blood Flow Index Evaluated by Ultrasonic Doppler under Intelligent Algorithm" was published in 2022. Journal: Comput Math Methods Med.

At 18-22 weeks of gestation, ultrasonic examination can screen out most fetal morphological and structural abnormalities [7, 8]. Arterial blood flow is one of the crucial parameters in physiopathological evaluation of the human body, which can show the benefits of fetal metabolism, and the distribution of blood flow velocity is of great significance in clinical measurement. Doppler ultrasound in medicine can be combined with intelligent algorithm to obtain the flow velocity of blood flow. In order to obtain Doppler flow echo signal, the physical model of carotid blood flow was first established by some studies [9]. There are some factors such as individual difference, noise interference, and poor acquisition of clinical data. Additionally, intelligent algorithms are used to get clearer test data [10, 11]. Ultrasonic Doppler can detect the indexes of umbilical arteries and veins of the fetus, and the ultrasonic Doppler frequency shift method can detect blood flow signal [7, 12–15]. The ultrasonic wave is accurately located by localization algorithm in ultrasonic localization. Compared with the traditional modified Newton algorithm, variable metric algorithm, and the fastest descent algorithm, the localization algorithm shows high accuracy. Additionally, the efficiency of image resolution in ultrasonic detection is improved by the adaptive algorithm. The empirical wavelet transform (EWT) algorithm refers to selecting a group of band-pass filters according to the signal spectrum characteristics, and the frequency range of the filter is determined. Line tracking technology is usually used in pulse radar speed measurement, which makes it difficult for the radar speed measurement system to track correctly [16, 17].

The accuracy of pulse radar Doppler speed measurement is improved. The acceleration to target and the phase compensation are particularly crucial. Time-frequency analysis method under the EWT algorithm was proposed. As ultrasonic measurement of UA was an important index of placental blood perfusion, the pulsatile index (PI), ratio of UA maximum systolic velocity of UA to the end of diastolic velocity or the resistance index (RI) to the fetal-placental blood circulation, and the resistance of the vascular bed were measured. Ultrasonic Doppler under the intelligent algorithm was employed to detect fetal umbilical arteriovenous blood flow index. The problem of FGR was discussed, and the value for the treatment of FGR was studied.

The article "Prediction of Fetal Growth Restriction for Fetal Umbilical Arterial/Venous Blood Flow Index Evaluated by Ultrasonic Doppler under Intelligent Algorithm" was published in 2022. Journal: Comput Math Methods Med.

## 2. Data and Methods

### 2.1. Clinical Data

In this study, 142 pregnant women who underwent prenatal ultrasonic examination in hospital from February 2018 to December 2020 were selected, and the gestational age was 22-40 weeks. The patients were performed with ultrasound examination method after adding intelligent algorithm. In addition, they were divided into FGR combination group and control group according to the ultrasound examination. The control group consisted of 102 patients with normal pregnancy, the mean age was 28.87 ± 3.72 years old, and the mean gestational age was 36.42 ± 2.67 weeks. The FGR group included 40 pregnant women with delayed fetal growth, the mean age was 29.31 ± 2.83 years old, and the mean gestational age was 36.71 ± 3.19 weeks. There was no significant difference in the generally clinical data between the two groups (*P* > 0.05), which indicated the comparability. The height, weight, age, gestational age, uterine height, and abdominal circumference of the fetus were recorded in detail. All the patients were excluded from contraindications to heparin use, and there was no abnormality in platelet coagulation function. All patients participated voluntarily and signed the informed consent forms and this study was approved by ethics committee of hospital.

The inclusion criteria of FGR were as follows: (I) women with singleton pregnancy; (II) women whose basic vital signs were stable, verbal, and conscious; (III) women in the age range of 18-70 years old; (IV) women with the slow growth of weight and uterine height; and (V) women whose fetal weight predicted by fetal growth diameters was 2 standard deviations that were lower than the estimated fetal weight of the same gestational age.

The exclusion criteria were as follows: (I) women with endogenous homogenous FGR caused by fetal chromosomal malformation; (II) women who were unwilling to join; (III) women with other systemic diseases; (IV) women who could not receive an ultrasound for their own reasons; and (V) women with incomplete clinical data.

### 2.2. Research Methods

#### 2.2.1. Ultrasound Method

The color Doppler ultrasound diagnostic instruments were adopted. The frequency range of abdominal convex array probe was 2.5-5.0 MHz. If FGR was found during the pregnancy examination, a conventional lateral position should be chosen for rest. Trace elements, nutrition, and oxygen absorption were given. 5000 IU of low molecular weight heparin was injected subcutaneously once a day, and one course of treatment was one week. Fetal weight was assessed after one week of treatment, and a postnatal or full-term fetal weight of less than 2.5 kg was diagnosed as growth restriction. Supine position was selected for the pregnant women. The fetus was examined in a quiet state without movement. Each standard section scan of two-dimensional ultrasound was used to exclude fetal malformation. Fetal parameters, including head circumference (HC), abdominal circumference (AC), and femur length (FL), were all measured routinely to determine placenta location. The fetal age and weight were estimated by observing whether the placenta was abnormal in the umbilical cord. When pulse Doppler was used to detect the UA blood flow index, the ultrasonic intensity and the average intensity of spatial peak time during imaging were lower than 100mw/cm^2^. The volume of the sample was 3 mm, and the angle between blood flow direction and sound velocity was less than 60 degrees. The index of blood flow = peak systolic rate (*S*) − end diastolic flow rate (*D*)/peak systolic flow rate (*S*). *S*/*D* = peak systolic flow rate (*S*)/end diastolic flow rate (*D*). PI = peak systolic flow rate (*S*)–end diastolic flow rate (*D*)/evaluation flow rate (*V*_mean_).

The article "Prediction of Fetal Growth Restriction for Fetal Umbilical Arterial/Venous Blood Flow Index Evaluated by Ultrasonic Doppler under Intelligent Algorithm" was published in 2022. Journal: Comput Math Methods Med.

#### 2.2.2. Ultrasound Basics

The frequency range of ultrasound in medicine is relatively limited, about 1 × 10^6^ − 1 × 10^7^ Hz. The ultrasonic wave propagates in the nonuniformity human body tissue. The reflection interface is different, the interface appears such physical phenomena as scattering, reflection, and refraction. The ability of the incoming sound wave produces different reflection coefficients at different interfaces. The larger the intrinsic impedance value of two adjacent tissues is, the greater the energy reflected by the interface will be, thus resulting in a smaller energy transmission. Part of the reason for ultrasonic weakness is mainly absorption by collagen. The relationship between attenuation coefficient and frequency is as follows.

(1) $$\begin{array}{c} W\left(\text{r}\right)=W_{0}{\text{e}}^{-{afo}^{r}}. \end{array}$$

In equation (1), *W*_0_ represents the initial sound pressure, *f*_0_ represents the acoustic frequency, and *a* represents the attenuation coefficient.

The schematic diagram of Doppler effect is shown in Figure 1.

Equation (2) shows the Doppler effect.

(2) $$\begin{array}{c} {\text{f}}_{d}={\text{f}}_{i}-{\text{f}}_{r}=\frac{2v\cos\partial }{c}f_{0}. \end{array}$$

In equation (2), *f*_*i*_ and *f*_*r*_ are the wave source and the received frequencies of the observation group. *f*_*d*_ represents the Doppler shift, and *v* means the velocity of the observer. The propagation velocity is generally 1,540 m/s. *α* shows the angle between the direction of propagation and the direction of motion of the observer. *f*_*d*_ represents the frequency of the wave source.

The article "Prediction of Fetal Growth Restriction for Fetal Umbilical Arterial/Venous Blood Flow Index Evaluated by Ultrasonic Doppler under Intelligent Algorithm" was published in 2022. Journal: Comput Math Methods Med.

Pulse Doppler ultrasound does not have the disadvantage of continuous Doppler range-free resolution. The Doppler echo signal within the target range can be precisely determined. Besides, some information about hemodynamics is also included in the Doppler information.

#### 2.2.3. The EWT Algorithm

EWT algorithm is a nonstationary signal processing algorithm. The advantages are mainly reflected in the number of single components, modal aliasing, and decomposition time. The main idea of the algorithm is dividing the Fourier spectrum adaptively. The constructed small filter banks are classified into corresponding intervals. Then, the amplitude and instantaneous frequency of the decomposed single component are obtained by the Hilbert variation.

The signal spectrum is classified into *N* consecutive parts. The Fourier spectrum of the signal is in the range [0, *π*]. The equation for each part is as follows.

(3) $$\begin{array}{c} \begin{array}{c} \Psi_{\text{n}}=\left[\omega_{n-1},\omega_{n}\right],\\ n=1,2,\cdots ,N\left(\omega_{0}=0,\omega_{N}=\pi \right). \end{array} \end{array}$$

Then, there is equation (4).

(4) $$\begin{array}{c} \cup_{\text{n}=1}^{N}\Psi =\left[0,\pi \right]. \end{array}$$

Boundary point *ω*_*n*_ and segment number *N* play a vital role in the adaptability of EWT algorithm. The selection flow chart of segment number *N* is shown in Figure 2. After *N* is determined, the first *N* maxima are selected from *T* maxima points. The positions in the corresponding spectrum are selected. Then, the median frequencies of the two maxima points are selected as boundary points.

After Ψ_n_ is identified, the extraction of single component requires adding wavelet function to construct empirical wavelet. Equation (5) shows the equation *ζ*_n_(*ω*) for empirical wavelet scale.

(5) $$\begin{array}{c} \zeta_{\text{n}}\left(\omega \right)=\left[0,\pi \right]\left\{\begin{array}{c} 1\left|\omega \right|\leq \omega_{\text{n}}-\lambda_{n}\\ \cos\left[\frac{\pi }{2}\beta \left(\frac{1}{2\lambda_{n}}\left(\left|\omega \right|‐\omega_{\text{n}}+\lambda_{n}\right)\right)\right]\\ \omega_{\text{n}}-\lambda_{n}\leq \left|\omega \right|\leq \omega_{\text{n}}+\lambda_{n}\\ 0\text{others} \end{array}\right.. \end{array}$$

The reconstruction equation for the original signal is as follows.

(6) $$\begin{array}{c} \text{x}\left(t\right)={M^{\chi }}_{\gamma }\left(0,\text{t}\right)*\zeta_{n}\left(t\right)+\overset{N}{\underset{n=1}{\sum }}{M^{\chi }}_{\gamma }\left(n,\text{t}\right)*\varepsilon_{n}\left(t\right). \end{array}$$

*M* ^*χ*^_*γ*_(0, t) represents the approximating function, and *M*^*χ*^_*γ*_(n, t) represents the detail function. ^∗^ means the convolution. Then, the *N* empirical mode equations are expressed as follows.

(7) $$\begin{array}{c} {\text{x}}_{0}\left(t\right)={M^{\chi }}_{\gamma }\left(0,\text{t}\right)*\zeta_{n}\left(t\right), \end{array}$$

(8) $$\begin{array}{c} {\text{x}}_{\text{k}}\left(t\right)={M^{\chi }}_{\gamma }\left(0,\text{t}\right)*\zeta_{n}\left(t\right)k=1,2,\cdots ,N-1. \end{array}$$

Normalized root mean square error is used for blood flow accuracy analysis, and equation (9) is used for calculation.

(9) $$\begin{array}{c} NRMSE=\frac{\sqrt{\sum_{k-1}^{e}\left(v\right.\left(c\right)-\bar{v}{\left(c\right)}^{2}}}{\sqrt{\sum_{k-1}^{e}\left(\bar{v}\right.{\left(c\right)}^{2}}}. \end{array}$$

In equation (9), *e* expresses the sample size, *v*(*c*) represents the estimated value of blood flow velocity, and$\bar{v}\left(c\right)$ shows the values of theoretical velocity at different points.

The article "Prediction of Fetal Growth Restriction for Fetal Umbilical Arterial/Venous Blood Flow Index Evaluated by Ultrasonic Doppler under Intelligent Algorithm" was published in 2022. Journal: Comput Math Methods Med.

#### 2.2.4. EWT Parameter Estimation Performance Analysis

The pulse emits cutting signal. The change of EWT in the estimation of FM signal parameter is 2. What the actual obtained is a group pf signal instantaneous frequency points *F* (*t*).

(10) $$\begin{array}{c} \text{F}\left(t\right)=F_{0}+\text{k}t+3k_{n}t^{2}+e\left(t\right). \end{array}$$

In equation (10), *e*(*t*) represents the frequency noise. EWT transform is a set of band-pass filters. Different instantaneous frequencies obtained by EWT transformation belong to different frequency ranges, and the method of frequency principal component extraction is employed to extract instantaneous frequency points in different frequency ranges. The frequency noise is only related to the signal-to-noise ratio (SNR). The least square method is used to evaluate the parameters. $\hat{\beta }$ expresses the linear unbiased estimation of *β*. Then, equation (11) is used to estimate the parameters.

(11) $$\begin{array}{c} {\text{e}}_{i}\left(t\right)=x_{0}+j{\text{k}}_{\text{i}}\left(t\right)=a_{\text{i}}\left(t\right)e^{j\theta_{i}\left(t\right)}. \end{array}$$

In equation (12), empirical model instantaneous frequency is regarded as the principal component of frequency.

(12) $$\begin{array}{c} {\left.K\left(t\right)=\arg\max a_{j}\left(t\right)\right|}_{t=\gamma }. \end{array}$$

#### 2.2.5. Statistical Method

SPSS 22.0 was employed for the test data. According to different situations, paired sample *t*-test was used to compare the changes of UA blood flow indexes before and after treatment. Besides, independent sample *t*-test was used for differences between the two groups, and analysis of variance was used for multiple data. When *P* < 0.05, it meant that the difference was statistically significant.

The article "Prediction of Fetal Growth Restriction for Fetal Umbilical Arterial/Venous Blood Flow Index Evaluated by Ultrasonic Doppler under Intelligent Algorithm" was published in 2022. Journal: Comput Math Methods Med.

## 3. Results

### 3.1. Statistics of the Clinical Data

Table 1 shows that there was no significant difference in the generally clinical data between the two groups (*P* > 0.05), indicating the comparability.

### 3.2. Time-Frequency Analysis Based on EWT

The main process of time-frequency analysis of EWT refers to using the algorithm to segment the Doppler blood flow echo signal adaptively and extracted the single component. The spectrum of the signal energy distribution in the time-frequency plane was obtained.  Figure 3 shows the segmentation of Fourier spectrum by EWT algorithm, presenting the single component Hilbert spectrum with Doppler shift.

### 3.3. Modal Function Instantaneous Frequency

Frequency patterns over different time periods were analyzed.  Figure 4 shows that the frequency principal component extracted by EWT method was little disturbed by noise. Most instantaneous frequencies were still distributed at both ends.

### 3.4. Comparison of Accuracy

The accuracy of blood flow velocity was calculated by normalized root mean square error. 50 samples were selected to estimate the velocity profile in different axial positions.  Figure 5 shows the comparison results with the accuracy of the traditional methods. The homogenization error of EWT was remarkably lower than that of short-time Fourier transform (STFT) algorithm (*P* < 0.05).

### 3.5. Ultrasonic Imaging

A 29-year-old female patient was selected. The history of chief complaint was that menopause was 26 + 3 weeks, and B-scan ultrasonography image showed that the fetus was 1 day younger than the gestational age. The auxiliary examination showed the stable vital signs, no obvious abnormality of the heart and lung, soft abdomen, no tenderness or rebound pain, and fetal heart beat 145 times/min. From the B-scan ultrasonography image, there were no abnormal amniotic fluid volumes, placenta maturity was 0 degree, and no other abnormal conditions were observed. After admission, the selected patient was given nutritional support and fetal heart monitoring, and the results showed that the pregnant woman was generally in good condition. Ultrasonic images of the pregnant woman were as follows.  Figure 6(a) shows the horizontal cross-section of the thalamus.  Figure 6(b) shows the head circumference and the dotted green line traced around the lateral edge of the skull.  Figure 6(c) shows color Doppler view of the front of the internal cervix.  Figure 6(d) shows the sagittal view of the internal cervix.  Figure 6(e) shows a cross-sectional sonogram of the hypothalamus. Besides, Figure 6(f) shows horizontal transverse view of the cerebellum.

The article "Prediction of Fetal Growth Restriction for Fetal Umbilical Arterial/Venous Blood Flow Index Evaluated by Ultrasonic Doppler under Intelligent Algorithm" was published in 2022. Journal: Comput Math Methods Med.

### 3.6. Comparison of Two Parameter Indexes

All parameters (inner diameter, cross-sectional area, mean blood flow velocity, and mean blood flow) were compared between the FGR group and control group.  Figure 7 shows the results that the inner diameter and cross-sectional area of FGR were notably smaller than those of the control group (*P* < 0.05). In the FGR group, there were no significant differences in mean blood flow and mean blood velocity compared with the control group (*P* > 0.05).

### 3.7. Comparison of Arterial Blood Flow Parameters

The RI and PI of arterial blood flow spectrum were compared between the FGR group and control group. In Figure 8, the results showed that there was no significant difference in RI between the two groups (*P* > 0.05). There was significant difference in PI between the two groups (*P* < 0.05). Additionally, PI of the FGR group was signally higher than that of the control group.

Arterial blood flow parameters, VS and VD, were compared and analyzed between the two groups. In Figure 9, the results showed that the FGR group was observably lower than the control group, with significant difference (*P* < 0.05).

## 4. Discussion

FGR is a relatively common obstetric complication. At present, the pathogenesis research has been developing continuously. The understanding of this disease also becomes profound [18, 19]. Ultrasonography is convenient and intuitive, which can monitor FGR by estimating the weight of the fetus and measure the UA blood flow index of the fetus [20]. Insulin helps to promote protein synthesis of amino acids in placental villi community and promote the synthesis of insulin-generating growth factor. Some studies showed that insulin and growth technique are markedly reduced in umbilical cord blood of FGR fetuses [21, 22]. In this study, the arterial blood flow indicators of the two groups of patients were compared and analyzed. The results revealed that the VS and VD in the FGR group were significantly lower than those in the control group, and the differences were statistically significant (*P* < 0.05). Ultrasound prediction FCR can measure the S/D value of fetal umbilical artery blood flow for many times, which is relatively random and noninvasive, and can provide important intrauterine development information for clinical practice.

With the increase of pregnant women's gestational weeks, venous blood flow parameters will also change to a certain extent. If the venous system is abnormal, the fetal heart and brain will have different degrees of damage, thus resulting in growth restriction and fetal prognosis dysplasia. [23]. Bakalis et al. [24] measured UA and fetal middle cerebral artery (MCA) of PI. In addition to maternal characteristics, medical history, and obstetric factors, measuring the cardiopulmonary resuscitation (CPR) was also important for the prediction of the pH of cord blood in the arteries and veins, after adjustment for variables affecting maternal characteristics and history. Both evaluation of fetal venous Doppler measurements in monochorionic twin pregnancy complicated with placental dysfunction and the relationship with academia at birth or intrauterine death were discussed by Liao et al. [28]. The ultraviolet (UV) Doppler parameter helps predict academia or intrauterine death in single birth and twins with placental insufficiency. EWT algorithm was introduced into Doppler ultrasound, and the imaging was set up according to the spectral characteristics of ultrasonic signal. The results showed that the frequency principal component extracted by EWT method was less disturbed by noise, which effectively evaluated fetal arteriovenous blood flow index and predicted FGR.

The article "Prediction of Fetal Growth Restriction for Fetal Umbilical Arterial/Venous Blood Flow Index Evaluated by Ultrasonic Doppler under Intelligent Algorithm" was published in 2022. Journal: Comput Math Methods Med.

## 5. Conclusion

The time-frequency analysis method based on EWT had low normalization error and high accuracy. The frequency principal component extracted by EWT method was less disturbed by noise. It could effectively evaluate fetal arteriovenous blood flow index, thus effectively predicting FGR. With the deep development of biomedicine, nonstationary signal is applied more and more in blood flow ultrasound. There are many kinds of intelligent algorithms. Therefore, in the future, other algorithms need investigating in the prediction of FGR by ultrasonic imaging. The limitation of this study was that the selected sample was relatively small, so it would increase the sample size, train the algorithm for many times, and analyze the signal stability in future.

## Figures and Tables

**Figure 1:** The schematic diagram of Doppler effect.

**Figure 2:** The flowchart of segment number selection.

**Figure 3:** The segmentation image of EWT.

**Figure 4:** Instantaneous frequency of EWT algorithm.

**Figure 5:** EWT error analysis. ^∗^ meant that there was significant difference, *P* < 0.05.

**Figure 6:** Color Doppler ultrasonography image.

**Figure 7:** Comparison of parameter indexes between the two groups. ^∗^ meant that there was significant difference, *P* < 0.05.

**Figure 8:** Comparison of the arterial blood flow parameters between the two groups. ^∗^ meant that there was significant difference, *P* < 0.05.

**Figure 9:** Comparison of blood flow parameters between the two groups. ^∗^ meant that there was significant difference, *P* < 0.05.

The article "Prediction of Fetal Growth Restriction for Fetal Umbilical Arterial/Venous Blood Flow Index Evaluated by Ultrasonic Doppler under Intelligent Algorithm" was published in 2022. Journal: Comput Math Methods Med.

**Table 1:** Comparison of general data between the two groups.

Group	Number of cases	Gestational age	Age (years old)	Height (cm)
FGR group	40	36.71 ± 3.19	29.31 ± 2.83	161.34 ± 2.23
Control group	102	36.42 ± 2.67	28.87 ± 3.72	162.34 ± 1.72
Statistical value		0.155	0.232	0.113
*P*		0.674	0.591	0.685

## Data Availability

The data used to support the findings of this study are available from the corresponding author upon request.
